The article "Inhibition of HMGB1-Induced Angiogenesis by Cilostazol via SIRT1 Activation in Synovial Fibroblasts from Rheumatoid Arthritis" was retracted in 2020. Reasons: errors in the images; concerns about the images.

# Inhibition of HMGB1-Induced Angiogenesis by Cilostazol via SIRT1 Activation in Synovial Fibroblasts from Rheumatoid Arthritis

**DOI:** 10.1371/journal.pone.0104743

**Published:** 2014-08-15

**Authors:** Hye Young Kim, So Youn Park, Sung Won Lee, Hye Rin Lee, Won Suk Lee, Byung Yong Rhim, Ki Whan Hong, Chi Dae Kim

**Affiliations:** 1 Medical Research Center for Ischemic Tissue Regeneration, Pusan National University, Yangsan, Gyeongnam, Republic of Korea; 2 Department of Pharmacology, School of Medicine, Pusan National University, Yangsan, Gyeongnam, Republic of Korea; 3 Department of Internal Medicine, College of Medicine, Dong-A University, Busan, Republic of Korea; Heart Research Institute, Australia

## Abstract

High mobility group box chromosomal protein 1 (HMGB-1) released from injured cells plays an important role in the development of arthritis. This study investigated the anti-angiogenic effects of cilostazol in collagen-induced arthritis (CIA) of mice, and the underlying mechanisms involved. The expressions of HIF-1α, VEGF, NF-κB p65 and SIRT1 in synovial fibroblasts obtained from rheumatoid arthritis (RA) patients were assessed by Western blotting, and *in vitro* and *in vivo* angiogenesis were analyzed. Tube formations by human microvascular endothelial cells (HMVECs) were significantly increased by direct exposure to HMGB1 or to conditioned medium derived from HMGB1-stimulated RA fibroblasts, and these increases were attenuated by cilostazol, the latter of which was blocked by sirtinol. HMGB1 increased the expression of HIF-1α and VEGF and concomitantly increased nuclear NF-κB p65 and DNA binding activity, but these effects of HMGB1 were inhibited by cilostazol. SIRT1 protein expression was time-dependently decreased (3–24 hr) by HMGB1, which was recovered by pretreatment with cilostazol (1–30 µM) or resveratrol, accompanying with increased SIRT1 deacetylase activity. In the tibiotarsal joint tissues of CIA mice treated with vehicle, HIF-1α- and VEGF-positive spots and CD31 staining were markedly exaggerated, whereas SIRT1 immunofluorescence was diminished. These variables were wholly reversed in cilostazol (30 mg/kg/day)-treated mice. Furthermore, number of blood vessels stained by von Willebrand factor antibody was significantly lower in cilostazol-treated CIA mice. Summarizing, cilostazol activated SIRT1 and inhibited NF-κB-mediated transcription, thereby suppressing the expression of HIF-1α and VEGF. In addition, cilostazol caused HIF-1α deacetylation by enhancing SIRT1 activity and reduced VEGF production, thereby had an anti-angiogenic effect *in vitro* studies and in CIA murine model.

## Introduction

Rheumatoid arthritis (RA) is characterized by uncontrolled hyperplastic synovium and inflammatory synovitis associated with the chronic production of proinflammatory cytokines and low oxygen tension. Hypoxia is a characteristic feature of RA synovitis, because limited vascular capacity makes it difficult to meet the greater oxygen demands of hyperplastic synovium present in active RA. Consequently, a state of chronic hypoxia is produced, which induces new vessel formation via the induction of pro-angiogenic mediators [1], [2]. Cellular response to hypoxia is driven by the hypoxia-inducible factor (HIF), which induces the expressions of large numbers of genes by interacting with specific promoter elements termed hypoxia-responsive elements [3]. Furthermore, the cytokines, IL-1β and TNF-α are known to increase HIF-1 protein accumulation in synovial fibroblasts (SF) by increasing its mRNA expression [4], [5]. High mobility group box chromosomal protein 1 (HMGB 1) levels are largely elevated in the synovial fluid samples of RA patients and potently trigger arthritis, and HMGB1 is reported to be actively secreted by macrophages or passively released by necrotic cells [6], [7]. Moreover, HMGB1 promotes the release of proinflammatory cytokines (TNF-α, IL-1β, and IL-6) from macrophages in synovial fluid [8], [9]. Hamada et al. [10] showed hypoxia increases extracellular HMGB-1, which localizes preferentially to regions of tissue hypoxia in arthritis lesions. In addition, these workers observed the attenuation of inflammatory pathology in a collagen-induced arthritis (CIA) mouse model after HMGB-1 neutralization, which suggests that tissue hypoxia and resultant extracellular HMGB-1 upregulation play important roles in the development of arthritis.

Several studies have shown that HMGB1 signals through RAGE or the toll-like receptors TLR2 and TLR4, and the activation of these receptors result in the activation of NF-κB, and thus, enhance the productions of proinflammatory cytokines and angiogenic factors in hematopoietic and endothelial cells, promoting inflammation [11]. Forsythe et al. [12] demonstrated the involvement of HIF-1 in the activation of VEGF transcription in hypoxic cells, and it was separately reported that HIF-1 binds to hypoxia-responsive element in the promoter region of the VEGF gene, and thus, upregulates VEGF expression [13].

Cilostazol is a phosphodiesterase type III inhibitor, and has been reported to exert potent anti-inflammatory effects. The anti-inflammatory actions of cilostazol suppress NAD(P)H oxidase-dependent superoxide formation, cytokine production (TNF-α, IL-1β etc.), and release of chemokines associated with reduced monocyte adhesion to HUVECs [14], [15]. As the underlying mechanisms involved, the anti-inflammatory actions of cilostazol were attributed to the cAMP-dependent protein kinase activation and to the suppression of NF-κB gene transcription [16], [17]. On the other hand, Lim et al. [18] proposed SIRT1 modulates cellular adaptation to hypoxia by targeting HIF-1α, and that SIRT1 directly deacetylates and inactivates HIF-1α. Furthermore, they revealed that SIRT1 prevents the secretion of VEGF in hypoxia, indicating SIRT1-induced deacetylation is responsible for inhibiting HIF-1 signaling.

Given that HIF-1α and VEGF signaling pathways play important roles in the regulation of angiogenesis, we hypothesized that cilostazol might regulate the HIF-1α and VEGF levels induced by HMGB1 in the SFs of RA. Thus, we investigated the signal pathways responsible for the inhibitory effect of cilostazol on synovial angiogenesis, and in particular, we attempted the following questions: (1) Does cilostazol suppress the expressions of HIF-1α and VEGF by inhibiting NF-κB activation? (2) Does cilostazol attenuate HIF-1α activity by enhancing SIRT1 expression and deacetylase activity? In addition, we sought to confirm that cilostazol inhibits HMVEC tube formation using an *in vitro* technique and by examining blood vessel formation *in vivo* in the arthritic synovia of CIA mice.

## Results

### Suppression by cilostazol of HMGB1-induced tube formation *in vitro*

We investigated whether the observed *in vitro* effect of HMGB1 on angiogenic processes is directly interfered with by cilostazol. When human microvascular endothelial cells (HMVECs) were directly exposed to HMGB1 (100 ng/ml) for 7 hr, tube formation significantly increased from 20.4±2.9 tubes/well (control) to 43.6±6.4 tubes/well (*P*<0.01), and pretreatment with 10 µM cilostazol reduced this HMGB1-stimulated tube formation to 18.5±3.5 tubes/well (*P*<0.05) (Fig. 1A and B).

**Figure 1:** Suppression of endothelial cell tube formation by cilostazol (CSZ). Photographs of tube formation induced by HMGB1 (100 ng/ml), which was applied directly to the HMVECs in the absence and the presence of 10 µM of cilostazol (A) and by conditioned medium (CM) derived from cultures of HMGB1 (100 ng/ml for 48 hr)-treated RA synovial fibroblasts (C). Diluted CM was added to the culture medium after adding HMVECs to Matrigel. Cultures were photographed after 9 hr (×100). (B and D) Quantitative analyses: Results are mean numbers ±SEM of tubes per well for 4–5 experiments. **P<0.01, ***P<0.001 vs. PBS (phosphate-buffered saline); ^##^ *P*<0.01, ^###^ *P*<0.001 vs. HMGB1 alone; ^†††^ *P*<0.001 vs. 10 µM cilostazol.

Based on the expectation that HMGB1-treated RA fibroblasts produce high levels of angiogenic factors, we compared HMVEC tube formation after treating them with conditioned medium (CM) derived from HMGB1 (100 ng/ml, for 48 hr)-stimulated RA fibroblasts or CM from vehicle-treated fibroblasts. CM was diluted 1∶5 in assay medium. Upon exposure of HMVECs to CM, the numbers of tubes formed increased significantly [(12.3±3.9 (vehicle group) to 34.5±4.0 tubes/well (HMGB1-treated), *P*<0.001)] (Fig. 1 Cb, c and Db, c). However, after pretreatment with 10 µM cilostazol, the number of tubes per well formed by these CM-treated HMVECs were significantly decreased (*P*<0.001) (Fig. 1Cd and Dd), and this decrease was prevented by pretreatment with sirtinol (20 µM, an inhibitor of SIRT1) (Fig. 1Ce and De). Additionally, pretreatment with YC-1 (30 µM, HIF-1α inhibitor) [19] inhibited HMGB1-induced tube formation, indicating that HIF-1α is involved in HMGB1-induced tube formation.

### Cilostazol suppressed the elevations of HIF-1α mRNA and protein expressions induced by HMGB1 in RA SFs

We also examined the effect of exogenous HMGB1 on HIF-1α mRNA and protein levels in RA SFs. As shown in Fig. 2A and B, the expressions of HIF-1α mRNA (*F*_3,12_ = 31.94, *P*<0.0001) and protein (*F*_3,12_ = 15.15, *P*<0.0002) were significantly elevated by treating SFs with 100–500 ng/ml of HMGB1 (*P*<0.001). Correspondingly, HIF-1α protein expression was time (3–24 hr)-dependently increased (*F*_4,15_ = 54.01, *P*<0.0001) by HMGB1 (100 ng/ml) (Fig. 2C).

**Figure 2:** Elevations of HIF-1α mRNA and protein expressions by HMGB1 and their inhibition by cilostazol. (A and B) Concentration-dependent HMGB1 (10–500 ng/ml)-induced increases in the mRNA and protein expressions of HIF-1α. (C) Time (3, 6, 12, and 24 hr)-dependent increases in HIF-1α protein levels in the presence of 100 ng/ml of HMGB1. (D) Concentration-dependent decrease of HMGB1 (100 ng/ml)-induced HIF-1α protein by cilostazol (CSZ; 1, 10 and 30 µM) and resveratrol (RES, 20 µM). (E and F) Reverse of cilostazol-induced decrease in HIF-1α mRNA (E) and protein (F) by KT5720 (1 µM; a cAMP-dependent protein kinase inhibitor), and significant suppression of HMGB1-induced HIF-1α mRNA by chetomin (10 nM, an inhibitor of hypoxia-inducible transcription) and by Bay11–7082 (1 µM, an inhibitor of I*κ*Bα phosphorylation). Results are the means ±SEM of 4–5 experiments. **P<0.01, ***P<0.001 vs. no treatment; ^#^ *P*<0.05, ^##^ *P*<0.01, ^###^ *P*<0.001 vs. HMGB1 alone; ^†††^ *P*<0.001 vs. 10 µM cilostazol.

To determine whether cilostazol suppresses HMGB1-induced upregulations of HIF-1α mRNA and protein, we pretreated RA SFs with cilostazol (1, 10 and 30 µM) for 4 hr prior to culturing them with 100 ng/ml HMGB1 for 12 hr. Increased HIF-1α protein expression by HMGB1was significantly reduced by cilostazol in a concentration-dependent manner [from 1.74±0.39 (100 ng/ml HMGB1) to 0.83±0.15 fold by cilostazol at 30 µM; *P*<0.001)]. Resveratrol (20 µM) had an effect similar to cilostazol on HIF-1α protein levels (Fig. 2D). Increased expression of HIF-1α mRNA by HMGB1 was also significantly inhibited by cilostazol (10 or 30 µM), and this was prevented by 1 µM of KT5720 (cAMP-dependent protein kinase inhibitor). Additionally, HIF-1α mRNA was significantly suppressed by pretreatment with chetomin (10 nM, *P*<0.001; an inhibitor of hypoxia-inducible transcription [20] as well as by Bay11–7082 [1 µM, *P*<0.001; an inhibitor of IκBα phosphorylation [21], pretreated for 30 min] (Fig. 2E). These results strongly suggest the involvement of NF-κB in the expression of HIF-1α mRNA and protein by HMGB1. Accordingly, HIF-1α protein level changes paralleled those of HIF-1α mRNA in response to HMGB1 and cilostazol (Fig. 2F). However, HIF-1β protein expression was not affected by HMGB1 (data not shown).

### Suppression by cilostazol of elevated VEGF mRNA and protein expression by HMGB1

HIF-1 was reported to bind to hypoxia-responsive element in the promoter region of the VEGF gene and to upregulate VEGF expression [12]. Thus, we first checked that VEGF mRNA and protein levels are increased in SF of RA in response to HMGB1. VEGF mRNA levels increased time (3–24 h)-dependently by over 2 fold at 12–24 hr (*F*_4,20_ = 13.73, *P*<0.0001) (Fig. 3A) and concentration-dependently to 1.90±0.26 fold (*F*_3,12_ = 16.24, *P*<0.0002) by 100 ng/ml HMGB1 (*P*<0.001) (Fig. 3B). Similarly, VEGF protein expression was also time- and concentration-dependently elevated by HMGB1 (Fig. 3C and D).

**Figure 3:** Suppression of HMGB1-induced elevations of VEGF mRNA and protein expressions by cilostazol. (A, B, C and D) Time- and concentration-dependent increases in VEGF mRNA and protein expressions stimulated by HMGB1. (E) Concentration-dependent suppression of HMGB1-stimulated VEGF mRNA expression by cilostazol (1–100 µM). (F) HMGB1-induced increase in VEGF releases and the attenuation of VEGF release by 10 µM cilostazol, by 30 µM YC-1 (HIF-1α inhibitor), and by 10 nM chetomin. The effect of cilostazol was blocked by KT5720 (KT, 1 µM) pretreatment. (G) Representative immunofluorescence photographs showing greater VEGF (+)-staining in HMGB1-treated synovial fibroblasts (24 hr), compared with control synovial fibroblasts. After treatment with cilostazol (10 µM), VEGF (+)-staining was obviously reduced. Results are expressed as means ±SEM of 4–5 experiments. **P<0.01, ***P<0.001 vs. no treatment; ^##^ *P*<0.01, ^###^ *P*<0.001 vs. 100 ng/ml HMGB1 alone; ^†††^ *P*<0.001 vs. 10 µM cilostazol.

It was determined whether the HMGB1-induced VEGF mRNA expression and protein release were suppressed by cilostazol. When cilostazol (1–100 µM) was co-treated with HMGB1 (100 ng/ml), HMGB1 (100 ng/ml)-induced increased VEGF mRNA expression was concentration-dependently reduced by cilostazol (1–100 µM) (*F*_5,18_ = 21.38, *P*<0.0001) (Fig. 3E). Furthermore, HMGB1-induced increased VEGF release (control, 159±12 ng/ml to 285±11 ng/ml by 100 ng/ml HMGB1) was significantly attenuated by 10 µM cilostazol (to 195±11 ng/ml, *P*<0.001), and this attenuation was wholly prevented by pretreatment with KT5720 (1 µM, *P*<0.001). In addition, pretreatment with either YC-1 (30 µM, a HIF-1α inhibitor) or chetomin (10 nM, an inhibitor of hypoxia-inducible transcription) significantly suppressed HMGB1-induced VEGF release, which strongly suggest involvement of HIF-1α in VEGF production (Fig. 3F).

These findings were further confirmed by an immunofluorescence study. When RA SFs were stained after being exposed to HMGB1 (100 ng/ml) for 24 hr, VEGF was largely expressed in the perinuclear region, but after pretreatment with cilostazol (10 µM) in the presence of HMGB1, this VEGF expression was greatly diminished (Fig. 3G). These results also suggest that HMGB1-induced increased VEGF release is reduced by cilostazol.

### Inhibition of NF-κB p65 activation by cilostazol

It has been previously demonstrated that NF-κB is a direct modulator of HIF-1α expression, and that HIF-1α promoter is responsive to selective NF-κB subunits [22]. Accordingly, we assessed the suppressive effect of cilostazol on NF-κB p65 activation in HMGB1-stimulated RA SFs. Stimulation of SFs with HMGB1 (10–500 ng/ml, for 30 min) caused concentration-dependent increase in expression of phosphorylated IκB, and nuclear NF-κB p65 expression was significantly increased [1.69±0.17 fold (*P*<0.001) by 100 ng/ml HMGB1] (Fig. 4A and B). Furthermore, the DNA binding activity of NF-κB p65 was concentration-dependently increased by HMGB1 (10–500 ng/ml), which was attenuated by pretreatment with glycyrrhizin (50 µM; an inhibitor of HMGB1 to DNA binding in cells) [23] and with Bay11–7082 (1 µM; an inhibitor of IκBα phosphorylation and NF-κB activation [21]) (Fig. 4C). Correspondingly, HMGB1 (100 ng/ml)-induced increase in expression of phosphorylated IκB [1.50±0.07 fold (*P*<0.001, N = 4)], nuclear translocation of NF-κB p65 and its DNA binding activity were all concentration-dependently repressed by cilostazol, respectively (Fig. 4D, E and F). Interestingly, the HMGB1-induced increase in phosphorylated IκBα, NF-κB nuclear translocation and DNA binding activity were significantly reduced by 20 µM of resveratrol, a known SIRT1 activator.

**Figure 4:** Inhibition of NF-κB p65 expression and activity by cilostazol. (A, B and C) HMGB1-induced increase in phosphorylated IκBα (A) and increase in the nuclear translocation of NF-κB (B) and DNA binding activity of NF-κB in synovial fibroblasts (C). These effects were inhibited by glycyrrhizin (50 µM, an inhibitor of HMGB1 binding to DNA) and by Bay11–7082 (1 µM). (D, E and F) Cilostazol (CSZ; 1, 10 and 30 µM) and resveratrol (RES; 20 µM) decreased phosphorylated IκBα (D), nuclear NF-κB (E) levels and DNA binding activity of NF-κB (F). (G, H) Suppression of HMGB1-stimulated production of proinflammatory cytokines, IL-6 and MCP-1, by cilostazol (10 µM) and the reversal of this suppression by KT5720 (1 µM) in cultured medium. Results are the means ±SEM of 3–4 experiments. *P<0.05, **P<0.01, ***P<0.001 vs. no treatment; ^#^ *P*<0.05, ^##^ *P*<0.01, ^###^ *P*<0.001 vs. HMGB1 alone; ^††^ *P*<0.01 vs. 10 µM cilostazol.

In line with these results, we verified the functional correlation between HMGB1 and proinflammatory cytokine productions in the absence or the presence of cilostazol by ELISA. As shown in Fig. 4 G and H, stimulation of RA SFs with HMGB1 (10–500 ng/ml) for 48 hr significantly increased the productions of IL-6 and MCP-1 (by 100 ng/ml HMGB1: IL-6 to 12.00±1.76 pg/ml, *P*<0.05 and MCP-1 to 28.03±3.52 pg/ml, *P*<0.05) in culture medium, and these increases were significantly suppressed by cilostazol pretreatment (10 µM). Furthermore, these suppressions by cilostazol were reversed by subsequent treatment with KT5720 (1 µM).

### Cilostazol increased SIRT1 expression and deacetylase activity

The effect of HMGB1 on the SIRT1 expression was explored in SFs. SIRT1 protein expression significantly decreased in a time (3–24 hr)-dependent manner after exposing RT SFs to HMGB1 (100 ng/ml) (*F*_4,15_ = 39.06, *P*<0.0001). When pretreated with cilostazol (1–30 µM) or resveratrol (20 µM) for 2 h prior to HMGB1 and cultured for 12 hr, HMGB1-induced decreases in SIRT1 protein expression were significantly restored by cilostazol (1.77±0.19 fold by 10 µM cilostazol, *P*<0.001) and by 20 µM resveratrol (1.66±0.27 fold, *P*<0.01) (Fig. 5A and B).

**Figure 5:** Increased SIRT1 expression and deacetylase activity by cilostazol. (A) Time (3–24 hr)-dependent decrease in SIRT1 protein expression after exposure to HMGB1 (100 ng/ml), and (B) recovery of reduced SIRT1 expression by cilostazol (1–30 µM) and by resveratrol (RES, 20 µM). (C) HMGB1-induced increase in H4 acetyl-k16 (H4 Ac-K16) immunoreactivity was decreased by cilostazol (10 and 30 µM) and resveratrol (RES, 20 µM). Cilostazol-induced decrease in H4 Ac-K16 was prevented by sirtinol (20 µM). (D) Analyses of SIRT1 knockout RA SFs compared with negative control cells. Cilostazol (10 µM) failed to induce expression of SIRT1 in RA SF cells transfected with SIRT1 siRNA oligonucleotide (100 nM) as contrasted to negative control. (E and F) Loss of the effect of cilostazol on the elevated expressions of p65 and acetyl (AC)-p65 induced by HMGB1 (100 ng/ml) in SIRT1 gene silenced fibroblasts, which contrasted to the effects of cilostazol in the negative control cells. Results are the means ±SEM of 4 experiments. **P<0.01, ***P<0.001 vs. no treatment or vehicle (Veh); ^##^ *P*<0.01, ^###^ *P*<0.001 vs. HMGB1; ^††^ *P*<0.01 vs. 10 µM cilostazol.

It has been previously reported by Lim et al. (18) that upregulation of SIRT1 leads to the deacetylation and inactivation of HIF-1α in hypoxia. We assessed SIRT1 activities in SFs by Western blots using an antibody specific for acetylated histone 4 lysine 16 residues (H4 Ac-k16). HMGB1significantly stimulated H4 Ac-k16 immunoreactivity (2.02±0.13 fold, *P*<0.001), which was significantly decreased by cilostazol (10 µM; to 1.29±0.22 fold, *P*<0.01 and 30 µM; to 1.08±0.22 fold, *P*<0.001) and by resveratrol (20 µM), and the effect of cilostazol was strongly blocked by sirtinol (20 µM, a SIRT1 inhibitor) (Fig. 5C). These results suggest that increased cilostazol-coupled SIRT1-mediated deacetylase activity prevented the HMGB1-induced acetylation of HIF-1α in SFs.

Since HMGB1-stimulated NF-κB activation was inhibited by cilostazol, we examined whether HMGB1-induced NF-κB p65 and acetyl-p65 expression were affected by cilostazol in the SIRT1 gene silenced RA SFs. With silencing of the SIRT1 gene (∼50% reduction in SIRT1 protein expression; Fig. 5D), cilostazol failed to reduce expression of NF-κB p65 and acetyl-p65 expression, whereas expression of NF-κB p65 and acetyl-p65 were decreased by cilostazol in cells transfected with scrambled siRNA duplex (negative control) (Fig. 5E, F), indicating the involvement of SIRT1 in the action mechanism of cilostazol.

### Immunohistochemistry and immunofluorescence studies in CIA mice

Histological study (H & E staining) revealed attenuated synovial tissue inflammation and reduced inflammatory cell infiltration in the tibiotarsal joints of mice treated with cilostazol (30 mg/kg/day). We adopted an immunofluorescence approach to determine whether cilostazol stimulates SIRT1 expression and suppresses the expressions of HIF-1α and VEGF in knee joints. In the vehicle-treated CIA mice, SIRT1 was expressed at low levels, whereas HIF-1α and VEGF were highly expressed. Interestingly, in mice treated with cilostazol (30 mg/kg/day), HIF-1α- and VEGF-positive spots were markedly attenuated, whereas SIRT1 immunofluorescence was markedly increased (Fig. 6A).

**Figure 6:** Immunohistochemistry (H & E and CD31) and immunofluorescence (SIRT1, HIF-1α and VEGF) assay. (A) Photographs showing SIRT1(+)-, HIF-1α (+)- and VEGF (+)-spots in joint sections of vehicle control and cilostazol (CSZ)-treated CIA mice. (B) Tibiotarsal joint tissue sections were stained with anti-CD31 antibody, and rabbit anti-human vWF (a marker of endothelial cells). Numbers of blood vessels/field and percentages of vWF stained area were analyzed in joint sections of CIA mice. Results are the means ±SEM of 4 experiments. *P<0.05, **P<0.01 vs. control; ^#^ *P*<0.05 vs. vehicle (Veh)-treated CIA mice. The pictures shown are representative of 4 experiments that produced similar results.

Additionally, CD31 expression, a marker of blood vessels, was high in vehicle-treated knee joints of CIA mice, and this was markedly attenuated in cilostazol-treated CIA mice as shown in control mice. To quantitatively analyze synovial angiogenesis, tibiotarsal joint tissue sections were stained with polyclonal rabbit anti-human von Willebrand factor (vWF, a marker of endothelial cells), and numbers of blood vessels were counted in joint sections. As shown in Fig. 6B, pronounced vWF staining area and vessel numbers were increased in the inflammatory synovial pannus areas of the paws of CIA mice treated with vehicle, and these were significantly diminished in cilostazol-treated CIA mice, indicating that cilostazol strongly attenuated angiogenesis in the synovium of the knee joints of CIA mice.

## Discussion

The major findings of the present study are that cilostazol inhibits *in vitro* tube formation by HMVECs and *in vivo* blood vessel formation with increased inflammatory severity in the arthritic synovium of CIA mice. The study confirms that the signaling pathways involved in HMGB1-induced HIF-1α expression and VEGF release involve NF-κB activation in RA SFs. Additionally, the study shows that cilostazol has two inhibitory effects, that is, (1) it inhibits HMGB1-induced increases in phosphorylated IκBα and the nuclear translocation of NF-κB, and thus suppresses HIF-1α expression, and (2) it inactivates HIF-1α by enhancing SIRT1 deacetylase activity, thereby suppressing VEGF expression at the mRNA and protein levels, and consequently inhibiting synovial angiogenesis (Fig. 7). Furthermore, our results provide first evidence that HMGB1 requires the upregulation of HIF-1α/VEGF for endothelial tube formation.

**Figure 7:** Hypothetical model. Scheme illustrating the dual effects of cilostazol, namely, (1) its inhibition of HMGB1-activated NF-κB nuclear translocation and subsequent HIF-1α expression, and (2) its inactivation of HIF-1α by increasing SIRT1 deacetylase activity in RA SFs. These effects lead to the down-regulation of VEGF and to the inhibition of synovial angiogenesis.

It has been established synovial inflammation is accompanied by fibroblast proliferation and neutrophil infiltration and by angiogenesis in RA patients. The uncontrolled proliferation of the synovial lining layer leads to microenvironmental changes resulting in hypoxic conditions [5], [16]. HMGB1 is either actively secreted by macrophages or passively released from necrotic cells [6], [7]. Furthermore, extracellular HMGB1 has been abundantly demonstrated in synovitis, that is, in the intra-articular fluids of RA patients and in animal models of arthritis [24]. In line with these results, Hamada et al. [10] have emphasized that concentration of HMGB1 significantly correlate with tissue hypoxia, indicating that extracellular HMGB1 plays a role as a coupling factor between hypoxia and inflammation in arthritis.

The cellular response to hypoxia is mainly driven by the transcription factor HIF [25]. Thus, in this study, measurement of HIF-1α protein in the presence of HMGB1 was considered as a marker of hypoxia. HIF-1 is a heterodimeric transcription factor and is composed of HIF-1α, which is oxygen regulated, and HIF-1β, which is expressed constitutively in the nucleus [26]. Our results show that exogenously applied HMGB1 markedly upregulated HIF-1α mRNA and protein levels, but not HIF-1β in RA SFs. Furthermore, these upregulations were significantly suppressed by cilostazol pretreatment, and these suppressions were reversed by KT5720, which concurs with the findings of Torii et al. [27]. In addition, VEGF mRNA and protein releases, which were increased time- and concentration-dependently by over 2 fold by HMGB1, were significantly attenuated by cilostazol. It was documented by Chun et al. [19] that YC-1 as a HIF-1α inhibitor blocked the induction of VEGF mRNAs. Considering that HMGB1-induced VEGF release and tube formation were inhibited by YC-1 and chetomin, an inhibitor of hypoxia-inducible transcription [20], it is likely considered that cilostazol-induced suppression of HMGB1-stimulated tube formation is ascribed to down-regulation of HIF-1α-linked VEGF release.

Recently, it was revealed NF-κB is a direct modulator of HIF-1α expression, and HIF-1α promoter is responsive to selective NF-κB subunits [22]. Furthermore, the classic hypoxia-responsive gene VEGF is present at high levels in the serum and synovial fluid of RA patients [28], [29]. In an experiment on IKK-2-deficient mice, NF-κB was proved to be required for HIF-1α protein accumulation, and the absence of IKK-2 resulted in defective induction of VEGF, a HIF-1 target [30]. Consistent with these reports, our results showed that HIF-1α mRNA was significantly suppressed by chetomin [20] and by Bay11–7082 (an inhibitor of IκBα phosphorylation [21]). These reported results indicate the involvements of hypoxia-induced transcription and NF-κB in the action of HMGB1. Thus, we examined the suppression of NF-κB p65 activation by cilostazol in HMGB1-stimulated RA SFs. Indeed, we found that the up-regulation phosphorylated IκBα and nuclear translocation of NF-κB p65 by HMGB1 were significantly attenuated by cilostazol and these were paralleled by a decrease in NF-κB p65 DNA binding activity. In view of several reports issued on the topic [22], [30], it appears likely that the down-regulations of HIF-1α and VEGF by cilostazol are due to reductions in NF-κB p65 activity.

Recently, Lim et al. [18] demonstrated that SIRT1 binds to, deacetylates and inactivates HIF-1α, and reported that during hypoxia, SIRT1 is downregulated due to diminished NAD^+^ levels, which allows the acetylation and activation of HIF-1α. Interestingly, we found SIRT1 protein expression was significantly decreased in a time (3–24 hr)-dependent manner after exposure to the HMGB1. The stabilization of HIF-1α protein is important in hypoxia, and hypoxia in turn increases extracellular HMGB-1 levels [9]. In the present study, we found that SIRT1 protein up-regulation by cilostazol coincided with enhanced SIRT1 deacetylase activity in SFs, as was reflected by reduced acetylation of the H4 Ac-k16, which support the notion that increased deacetylation of HIF-1α by cilostazol is responsible for the reduced induction of VEGF. Importantly, in the synovial fibroblasts transfected with SIRT1 SiRNA, cilostazol failed to reduce the expression of NF-κB p65 and acetyl-p65, as contrasted to the negative control cells (transfected with scrambled siRNA duplex). These findings strongly suggest that inhibition of NF-κB p65 acetylation by deacetylase activity of SIRT1 is involved in the action mechanism of cilostazol.

As was expected, in the tibiotarsal joint tissues of CIA mice, SIRT1 expression was markedly diminished and in contrast HIF-1α and VEGF were highly up-regulated in concert with CD31. Furthermore, these angiogenic factors were substantially diminished by cilostazol (30 mg/kg/day) and in contrast SIRT1 immunofluorescence was markedly increased. In line with these observations, pronounced vWF staining and increased numbers of vessels, observed in the inflammatory synovial pannus area of CIA mouse, were significantly diminished by cilostazol, which reflects its anti-angiogenic effect.

Summarizing, this study shows cilostazol activates SIRT1, and thus, elicits dual effects in RA SFs, that is, (1) it inhibits NF-κB-mediated transcription, which suggests the suppressions of HIF-1α and VEGF, and (2) it increases HIF-1α deacetylation by enhancing SIRT1 activity, which further blocks VEGF expression and leads to the inhibition of synovial angiogenesis.

## Materials and Methods

### Animals

All the animals procedures were confirmed in accordance with the Guide for the Care and Use of Laboratory Animals published by the US National Institutes of Health (NIH Publication No. 85-23, revised 1996), and experimental protocols were approved by the Pusan National University Institutional Animal Care and Use Committee. Male DBA/1J mice (aged 8–12 weeks) were purchased from Japan SLC, Inc. (Shizuoka, Japan). All animals were housed in a temperature and humidity controlled animal facility under a 12-h light-dark cycle.

### Collagen-induced arthritis (CIA)

CIA was induced in DBA-1 mice as previously described by Park et al. [17]. Briefly, 100 µg of bovine type II collagen (Chondrex, Redmond, WA) dissolved in 0.1 M acetic acid was emulsified with an equal volume of Freund's complete adjuvant (Sigma, St Louis, MO) and administered intradermally at the base of the tails of DBA/1J mice. On day 18 after the first injection, a booster emulsion prepared with type II collagen and Freund's incomplete adjuvant (Sigma) was intradermally administered near the primary injection site. Using the same protocol, adjuvant-treated littermates received phosphate-buffered saline (PBS) in place of type II collagen and served as controls. Cilostazol (30 mg/kg/day) was administered from the day after the booster injection. Thirty-five days after implantation, mice were sacrificed by cervical dislocation.

### Cell preparations

#### Synovial fibroblasts

Synovial fluid samples were obtained from the knees of RA patients, who fulfilled the 1987 revised criteria of the American College of Rheumatology (formerly, the American Rheumatism Association), at the time of therapeutic arthrocentesis. All patients who attended a rheumatology clinic provided informed consent, and the ethics committee of Dong-A University Hospital (Busan, Korea) approved the study protocol. Synovial cells were obtained as described by Neidhart et al. [31]. Briefly, synovial fluid samples were centrifuged at 450×g for 30 min, and pellets were resuspended in Dulbecco's modified Eagle's medium (DMEM) containing 10% fetal bovine serum (FBS), and incubated for 24 hr at 37°C. Non-adherent cells were removed by washing, and medium was changed daily for 3 days. Remaining adherent round monocytes and spindle-shaped fibroblast-like cells were cultured for 2 additional weeks in a flask. The adherent round monocytes that attached to the flask were resistant to trypsinization. In contrast, the spindle-shaped fibroblast-like synovial cells were easily collected by trypsinization. These cells were removed and placed in a new culture flask, and used for experiments at passages 4 to 6.

#### Endothelial cells

Human microvascular endothelial cells (HMVECs) (Lonza, Waterville, Inc, California) were cultured in endothelial cell basal media-2 (EGM-2) (Bullet kit medium; Clonetics, BioWhittaker, San Diego, CA). HMVECs were grown to confluence at 37°C in 5% CO2 and used for experiments before passage 6.

### Reverse transcription–polymerase chain reaction (PCR)

Total RNA was extracted from synovial fibroblast-like cells using TRIzol reagent (Invitrogen, San Diego, CA). The PCR primers used were as follows: for HIF-1α, 5′-AAATCTCCGTCCCTCAACCT-3′ (sense), 5′-GAAAACTTGGCAACCTTGGA-3′ (antisense), and VEGF, 5′-ATCTGCATGGTGATGTTGGA-3′ (sense), 5′-AAGGAGGAGGGCAGAATCAT-3′ (antisense). PCR was conducted using cycles consisting of 95 °C for 1 minute followed by hybridization at 56 °C for 1 minute and an elongation step at 72 °C for 1 minute. Relative mRNA expressions were normalized versus GAPDH mRNA, the levels of which were not altered by treatments. The mRNA expressions of cells treated with vehicle alone were set arbitrarily at 1.

### Western blot analysis

Protein (30 µg) samples were loaded onto 10% SDS-polyacrylamide electrophoresis gels and transferred to nitrocellulose membranes (Amersham Biosciences, Inc., Piscataway, NJ). Blocked membranes were then incubated with antibodies for HIF-1α (Cell Signaling Technology, Danvers), NF-κB p65, IκB-α (Santa Cruz Biotechnology, Inc. Santa Cruz), and acetylated histone 4 lysine 16 residue (H4-k16Ac) antibody (Santa Cruz Biotechnology). Immunoreactive bands were visualized using the chemiluminescent reagent in the Supersignal West Dura Extended Duration Substrate Kit (Pierce Chemical, Rockford, IL). Band signals were quantified using a GS-710 calibrated imaging densitometer (Bio-Rad, Hercules, CA). Results are expressed as relative densities.

### Tissue preparation and conventional histological analysis

Whole knee joints from mice were dissected and fixed for 1 day in 4% paraformaldehyde, decalcified in 10% EDTA, dehydrated, and embedded in paraffin blocks. Blocks (6-µm thick) were cut and stained with hematoxylin and eosin (H&E) for the assessment of synovial inflammation and bone erosion.

### Immunocytochemistry and Immunofluorescence assays

For immunocytochemistry, synovial tissues were fixed with 4% paraformaldehyde, permeabilized with 0.2% Triton X-100, incubated with anti-CD31 antibody for 1 hr, and then with FITC- and Cy3-conjugated secondary antibodies for 30 min. Fluorescent images were obtained using a confocal microscope (OLYMPUS FV-1000, Tokyo, Japan).

In immunofluorescence experiments, preparations were incubated for 1 hr at room temperature with anti-VEGF (Santa Cruz Biotechnology, Inc), anti-HIF-1α (Cell signaling Technology), antibodies against SIRT1 (Covance, Emeryville, CA) and anti-von Willebrand factor (vWF) antibodies. After washing, sections were incubated with a secondary antibody solution for 30 min at room temperature, and mounted using Vectashield mounting medium (Vector Laboratories, Inc.). Fluorescence was detected using a fluorescence microscope (Axiovert 200, Carl Zeiss, Oberkochem, Germany).

### Enzyme-linked immunosorbent assay

The levels of IL-6, and MCP-1 in culture supernatants were measured using an ELISA kits (Assay Design Inc., Ann Arbor, MI), according to the manufacturer's instructions.

### NF-κB transcription factor assay

To measure levels of NF-κB transcription factor in nuclear extracts, cell lysates were extracted using a nuclear extraction kit (Chemicon International, Temecula, CA). NF-κB p65 DNA binding activities were measured using a colorimetric NF-κB p65 transcription factor assay kit (Rockland Immunochemicals, Gilbertsville, PA), according to the manufacturer's instructions.

### Tube formation assay

For obtaining the conditioned medium (CM), RA SF were plated in DMEM containing 1% FBS. The next day, cells were treated with vehicle or HMGB1 (100 ng/ml) for 48 hr. Culture media (CM) were collected and stored at −20°C until required. To perform the tube formation assay, Matrigel Matrix (BD Biosciences, Sanjose, CA) was polymerized for 30 min at 37°C in 48 well plates. HMVECs were then removed from culture by trypsinization and suspended in basal medium (EBM containing 1% FBS). They were then plated onto Matrigel layers, and placed in HMGB1-containing medium or CM (diluted 1∶5 in assay medium) at 37°C, and 7∼9 hr later cultures were photographed (×100).

### Drugs

Cilostazol (OPC-13013) [6-[4-(1-cyclohexyl-1H-tetrazol-5-yl)butoxy]-3,4-dihydro-2-(1H)-quinolinone] was donated by Otsuka Pharmaceutical Co. Ltd. (Tokushima, Japan), and was dissolved in dimethyl sulfoxide to produce a 10 mM stock solution. Recombinant Human HMGB1 was obtained from R&D Systems (Minneapolis, MN), and chetomin from Enzo Life Sciences (Plymouth Meeting, PA; purity >98% by HPLC analysis). BAY11-7082 [(*E*)3-[(4-methylphenyl)-sulfonyl]-2-propenenitrile], KT5720, resveratrol, and glycyrrhizin (a glycoconjugated triterpene produced by Glycyrrhiza glabra (licorice) from Sigma (St. Louis, MO). YC-1 [3-(5′-hydroxymethyl-2′-furyl)-1-benzylindazole] was from Cayman Chemical (Ann Arbor, MI] and dissolved in 1% DMSO. CD31 polyclonal antibody (1∶2,000 dilution; Abcam, Cambridge, UK) and monoclonal anti-vWF antibodies (1∶300 dilution; Dako, Glostrup, Denmark) were used to evaluate blood vessel numbers.

### Statistical analysis

Results are expressed as means ±SEM. The significances of results were analyzed by one-way analysis of variance (ANOVA) followed by Tukey's multiple comparison test. The Student's *t*-test was used to determine the significances of differences between treated and untreated groups. Statistical significance was accepted for *P* values <0.05.
